RETRACTED

# An Intelligent and Fast Dance Action Recognition Model Using Two-Dimensional Convolution Network Method

**DOI:** 10.1155/2022/4713643

**Published:** 2022-07-09

**Authors:** Shuai Zhang

**Affiliations:** School of Music, Shanxi Normal University, Taiyuan 030032, China

## Abstract

In the field of computer vision, action recognition is a very difficult topic to study. This paper suggests a dance movement recognition method based on DL network in accordance with the characteristics of dance movements. The backbone network in this study is a thin network called Mobile Net. The two-dimensional convolution network, which can only extract spatial features, can extract and fuse time domain features and use them for dance movement recognition by combining the time domain modelling strategy of time domain feature transfer between convolution layers. It uses fewer network parameters and less computation than the original multitarget detection model. Using the clustering method to preset the prior frames of human detection with various sizes and numbers also enhances the model's performance. Finally, the experimental findings demonstrate that the algorithm suggested in this paper outperforms the Incision v3 algorithm in F1 by 9.87 percent and outperforms the traditional CNN algorithm in identification accuracy by 6.51 percent and 10.76 percent, respectively. It is evident that the algorithm used in this paper reduces running time and, to a certain extent, improves the accuracy of dance movement recognition. For related research, it offers some references.

## 1. Introduction

Action recognition, which is a crucial component of video analysis, has been extremely important in many crucial fields. The video field has also adopted DL to deal with video action recognition tasks due to the performance of DL (deep learning) [1, 2] in recent years, which significantly outperforms the manual features in image classification, object detection, and semantic segmentation. The primary goal of the research, which is significant for DL applications, is to learn about and comprehend the behaviours and actions of the characters by computer processing and analysis of the photos or videos taken with a camera. Current computer research is focused heavily on body action recognition in video. Through a variety of image processing [3], segmentation [4], and classification technologies [5], it aims to extract and analyse motion from videos in order to judge the actions of the characters in the footage and gather useful data. Applications for it are extremely varied. Due to dance's high level of complexity and self-occlusion, there are not many studies that combine video-based action recognition technology with dance videos. As a result, more work needs to be done in this area. In the process of teaching dance movement, students or instructors can standardise the movements using the outcomes of human movement recognition; for minority dances, human body movement recognition can also obtain and save the essential information of dance movements, lowering the risk of dance disappearing during the inheritance process. The study of dance movement identification therefore has some application.

RETRACTED

At present, the mature DL network structures in the image field include AlexNet structure, VGGNet structure, GoogLeNet structure, and ResNet structure. Traditional body action recognition is mainly based on RGB images or videos, but due to the influence of scale, illumination changes, and background noise, the effect is not satisfactory. In recent years, thanks to the development of depth sensors and the maturity of key point detection algorithms of human bones, more and more researches focus on the action recognition algorithms based on key points of bones and begin to use graph convolution to model and analyse human bones. Compared with images, the biggest difference between videos is that they contain information in time domain. How to effectively use the information in time domain is a very important research point in the task of video action recognition. The key of video action recognition is to preprocess the original video image reasonably, then extract the features of the video image, and describe and classify them. CNN (convolutional neural network) [6, 7] is the most commonly used DL network in the field of image processing. DL is a data-driven method, so a lot of labelled data is needed in the training process [8]. In recent years, researchers have paid more attention to the video field, and a large number of data sets have been put forward, which further promotes the role of DL in video analysis. Based on DL technology, this paper makes an in-depth exploration of dance movement recognition methods. Its innovations are as follows:

① In this paper, Mobile Net, a lightweight network, is used as the backbone network. By combining the time domain modelling strategy of time domain feature transfer between convolution layers, the two-dimensional convolution network, which can only extract spatial features, can extract and fuse time domain features and use it for dance action recognition. At the same time, using multiple small convolution kernels instead of large convolution kernels increases the nonlinear expression ability of the model. On the input data, the improved 3D network is trained by using different combinations of various data, and the optimal input data format is determined by analysing the experimental results of different groups.
② In this paper, the identification and classification results are obtained by two-layer full connection and Softmax classifier, and the scale invariant feature descriptor and the moving history edge image are used as auxiliary features for regularization. In addition, the Fusion Inception network, which can fuse the convolution features of each layer, is used to extract the image features, and a branch design is adopted in the prediction module. Meanwhile, the convolution network model is trained by using classification and regression errors. Simulation results show that the method proposed in this paper has higher identification accuracy and faster running speed.

RETRACTED

This paper's main argument is the identification of dance movements. How the paper's chapters are organised is as follows: Introduction is covered in chapter one. The research topic, research history, and significance of this paper are presented in this section. This paper provides a brief overview of the research innovation and paper's organisational structure. A related chapter is the second one. This section explains the relevant research literature and the current state of the field. The related foundation and theory of DL are briefly introduced in the third chapter, and the issue of action recognition is covered in detail from two angles: feature extraction method and classifier. Then, in order to address the shortcomings of the current action recognition methods, a dance action recognition method based on DL is suggested, along with a detailed description of the implementation procedure. The experimental section is in chapter four. The summary and prospect chapter is the fifth. The work of this paper is summarised in this chapter, which also suggests some improvements and lines of inquiry for future study.

## 2. Related Work

Wang H et al. established a body detection model based on the YOLONano network to locate the position of the body in the picture. Based on the YOLONano multitarget detection model, a human body detection model is established by correcting the number of network output channels while retaining the category of people. Compared with the original multitarget detection model, the network parameters and computational complexity are reduced [9]. Ma et al. proposed a strategy to train the network with balanced loss instead of cross-entropy classification loss for the imbalance of head pose angle class samples [10]. Aiming at the problem of combining action recognition with dance videos, Kavi et al. focused on feature extraction, representation, and action recognition methods based on dance videos [11]. Murtaza et al. improved the traditional DL network to meet the needs of rapid and accurate recognition of video actions on the Internet and constructed a two-way convolution network in time domain and space domain [12]. Cai et al. mainly studied the recognition of body actions in action videos using techniques such as image preprocessing, 3D Zernike moments, building codebooks, and SVM [13]. Aiming at the real-time requirements of actual natural human-computer interaction, Yao et al. proposed a new human-computer interaction method that integrates video key frame extraction and human partial action recognition [14]. In order to improve the performance of specific dance action recognition in machine vision, Li et al. designed a specific dance action recognition method based on global context [15]. Li et al. proposed a dance action detection method based on gesture recognition [16]. Nazir et al. proposed a 3D convolutional network based on visual attribute mining, using 3D convolutional network to learn the expression of video and then recognise the action [17]. This method addresses the misclassification problem of existing networks on videos with similar spatial and temporal patterns. In order to realise the accurate detection and recognition of body actions, Xu and Yan proposed a deep information recognition method of body actions based on machine learning [18]. The method constructs a 3D image acquisition model of human motion and establishes a surface structure reconstruction model for 3D reconstructed images of human motion.

RETRACTED

This paper method uses the lightweight network Mobile Net as the backbone network and combines the temporal modelling strategy of temporal feature transfer between convolutional layers, so that the two-dimensional convolutional network that can only extract spatial features can extract and fuse temporal features, which is used for dance movement recognition task. At the same time, by combining the key point information of the bones, the relative positions of human joint points, joint point angles, and limb length ratio fusion features are selected to classify the movements in the dance scene, and the automatic action detection method of the residual block is used to realise the dance of complex dance scenes. Studies have shown that the method in this paper can effectively identify dance movements and then perform movement corrections for dancers.

## 3. Methodology

### 3.1. An Overview of Dance Movement Recognition Methods

Data collection and preprocessing, human feature extraction and construction, and motion recognition are crucial elements of body behaviour recognition. The primary factor in determining whether or not to recognise human motion is the development of body features. The feature extraction and construction techniques currently in use, however, are typically not accurate enough. CNN has a wide range of application scenarios in computer vision, natural language processing, and other fields, and its related technologies are becoming more and more mature and are often used in tasks such as classification, recognition, segmentation, and translation. Multichannel CNN-based DL methods are a class of widely used methods in video action recognition tasks. This kind of method firstly learns the features of multiple domains or multiple modalities and then uses feature fusion to effectively aggregate the information of multiple domains or multiple modalities. The feature map of the same layer convolution of CNN is transferred in the temporal domain to model the image frame sequence in the temporal domain [19]. Through the way that the convolutional layer of CNN exchanges some feature maps at the same layer at different times, CNN can not only directly extract the temporal information of image sequences to a certain extent, but also realise the fusion of temporal and spatial domain features naturally, and this method does not introduce extracomputation. By mapping the data into a low-dimensional Euclidean space, CNNs can be effectively employed to extract effective features. After acquiring the features, the network can be used to perform the video action recognition task end-to-end, or these features can be input into the classifier as a representation of a video to identify the video and then understand the human behaviour in the video, and based on the function of the system, it makes corresponding decisions [20]. In the video action recognition task, DL architectures based on multichannel NN (neural network) and 3D CNN have achieved good performance so far. The convolution operation in CNN refers to multiplying the input neurons by a specific set of weights. This set of weights is called a filter. This set of filters performs a sliding window operation on the image so that the CNN can learn from the image feature.

RETRACTED

Compared with DL algorithms based on images or videos, action recognition algorithms based on skeleton key points are more robust to scale, illumination changes, and background noise and are immune to changes in camera perspective, rotation, and movement speed of the human body [21]. This makes the action recognition algorithm based on skeletal key points perform better on some data sets. For spatial NN, the input is the RGB data of some frames in the video; for temporal NN, the input is the data of continuous optical flow field, and we can also input the optical flow data as a kind of image-like RGB format data to the network to train. After the two NNs are trained in the previous layers, each of them finally passes through a Softmax layer, and then the results of Softmax are weighted and added as a feature of the final entire video. This method has a simple structure, is easy to train, and achieves good results. Body action recognition network is a recognition algorithm based on PAFs algorithm, which can accurately identify the key points and actions of human skeleton in images. The main process is to extract features through the first 10 layers of the VGG19 network and send them into the key point heat map branch and limb vector branch to realise the recognition of body actions. The NN model is shown in Figure 1.

Traditional NN is really only suitable for structured data, such as images and text sequences, and graph-structured data is not suitable. To solve this problem, graph CNNs are proposed, which mainly focus on how to construct DL models on graphs. Multichannel NN is a class of widely used network frameworks in video action recognition tasks. It effectively aggregates the information of multiple domains by learning the features of multiple domains separately and then performing feature fusion. However, there is a lot of contextual information in the video, including the position information of the subject acting in the video, the information of the objects around the subject, and the background information. These kinds of information can be regarded as a kind of semantic information, which can provide effective help for the video action recognition task. With the development of technology, lightweight networks have begun to rise. A series of lightweight networks represented by Mobile Net not only maintains high classification performance, but also makes full use of grouped convolution and 1 × 1 convolution technology to greatly reduce the model. The amount of parameters makes it possible to perform real-time operations on many tasks. In action recognition research, the first thing to do is usually feature extraction. The hand-designed feature-based method employs an ingeniously designed underlying feature extraction algorithm to effectively obtain the structured information in the video frame and uses the machine learning method to train the model on this information to classify the video. Since the number of handcrafted features is not fixed, the features need to be further aggregated and then input into the machine learning model.

### 3.2. Dance Action Recognition Model Based on DL Network

DL-based dance action recognition algorithms usually include the following three steps. (1) Extract features from images or videos. (2) Model the action of the extracted features. (3) Match the modelled high-level features with action categories. The dance movements in dance performances are often too complex, and it is difficult to use traditional single movement features to characterise complex dance movements due to the influence of factors such as the speed of the individual's performance and the difference in acquisition speed. Therefore, the difficulty of dance action recognition lies in how to extract effective features to accurately characterise the dance actions in dance videos. First, the input image is cropped to 368^*∗*^368 size and the human body key points are recognised by the input pose recognition network. Then, the human body region is detected by the residual network according to the contour value of the human body key point. Finally, by fusing the key point feature classification and image classification, the classification of dance movements can be realised. The dance action recognition process based on DL network is shown in Figure 2.

RETRACTED

The skeleton key point sequence provides more comprehensive human body structure information. In the form of two-dimensional coordinates, the dynamic skeleton of the human body can be naturally represented by the human skeleton key points of consecutive multiple frames, and with the help of the additional geometry provided by the depth image with depth information, NN can more easily model the connections between human joints. The architecture of the Mobile Net network is shown in Table 1.

Preprocessing includes background subtraction and median filtering. The background subtraction is used to extract the foreground and separate the human motion area. The median filtering is used to filter out the noise in the image to reduce the influence on edge features. The pixels in the image have a clear relationship between the upper, lower, left, and right positions, and the words in the sentences have a clear sequence structure, which can be converted into low-dimensional Euclidean structured data and input into NN for feature extraction and calculation. For the task of classification and recognition, it is of great significance to accurately grasp the inherent laws of the data, express the data effectively, and carry out feature classification or regression for subsequent machine learning algorithms.

On the basis of the cross-entropy loss, the balance loss can adjust the loss by weighting the function of ${\hat{y}}_{k}$, and its expression is as follows:

(1) $$\begin{array}{c} \text{BL}\left(y,\hat{y}\right)=-\sum_{k=1}^{N}t_{k}\frac{1}{\gamma +1}{\left(1-{\hat{y}}_{k}\right)}^{\gamma }\log\;{\hat{y}}_{k}. \end{array}$$

In the above formula, *γ* is a nonnegative regulator. During network training, the calculation method of the total loss function of each channel is the same, which consists of the classification loss BL and the regression loss MSE (mean square error). The total loss calculation formula is as follows:

(2) $$\begin{array}{c} \text{ML}=\text{BL}\left(y,\hat{y}\right)+\alpha \text{MSE}\left(y{}^{\prime }-\hat{y}{}^{\prime }\right). \end{array}$$

In the above formula, *α* is a weight coefficient that adjusts the proportion of classification loss and regression loss. The gesture recognition network is used for iterative prediction, and the calculation method of the prediction is as follows:

(3) $$\begin{array}{c} S^{I}=\rho^{I}\left(F,S^{I-1},L^{I-1}\right),\;\forall t\geq 2,\\ L{}^{\prime }=\Phi^{t}\left(F,S^{t-1},L^{t-1}\right),\;\forall t\geq 2. \end{array}$$

Add a loss function in the calculation process, as shown in the formula:

(4) $$\begin{array}{c} f=\sum_{t=1}^{T}\left(f_{x}^{t}+f_{l}^{t}\right),\\ f_{s}^{t}=\sum_{j=1}^{J}\sum_{p}W\left(p\right)•{\left\|S_{j}^{I}\left(p\right)-S_{j}^{\cdot }\left(p\right)\right\|}_{2}^{2},\\ f_{L}^{t}=\sum_{c=1}^{C}\sum_{p}W\left(p\right)•{\left\|S_{c}^{I}\left(p\right)-S_{c}^{\cdot }\left(p\right)\right\|}_{2}^{2}. \end{array}$$

In the formula, *f*_*s*_^*t*^ and *f*_*l*_^*t*^ represent the key point confidence map and the predicted value of PAFs, respectively; *S*_*j*_^•^ and *L*_*c*_^•^ represent the key point confidence map and the true value of PAFs, respectively. The Softmax cross-entropy function is chosen in this paper, and its form is as follows:

(5) $$\begin{array}{c} \text{loss}=\sum_{i}\sum_{c}y_{c}\cdot \;\log\left(y{\text{pred}}_{c}\right). \end{array}$$

Among them, *c* represents the category of classification, and when the output result is consistent with the actual category, *y*_*c*_=1. The purpose of image thresholding is to obtain binary images of moving images. Generally, the threshold can be written as follows:

(6) $$\begin{array}{c} T=T\left[x,y,f\left(x,y\right),p\left(x,y\right)\right]. \end{array}$$

In the formula, *f*(*x*, *y*) is the gray value at the pixel point (*x*, *y*); *p*(*x*, *y*) is the gray gradient function of the point. The binarized image can be obtained by using the above formula. For an image sequence, the formula for calculating Zemike moments is as follows:

(7) $$\begin{array}{c} A_{nm\mu y}=\frac{n+1}{\pi }\sum_{i=1}^{\text{images}}\sum_{x}\sum_{y}U\left(i,\mu ,\gamma \right)\left[V_{nm}\left(r,\theta \right)\right]P_{i}\left(x,y\right). \end{array}$$

In the formula, images represent the number of images in the whole sequence; *U*(*i*, *μ*, *γ*) is the introduced third dimension:

(8) $$\begin{array}{c} U\left(i,\mu ,\gamma \right)={\left(\bar{x_{i}}-\bar{x_{i-1}}\right)}^{\mu }{\left(\bar{y_{i}}-\bar{y_{i-1}}\right)}^{\gamma }. \end{array}$$

In the formula, $\bar{x_{i}}$ represents the center of gravity of the current image; $\bar{y_{i-1}}$ represents the center of gravity of the previous image.

RETRACTED

This paper takes a high-resolution subnet as the first stage. After each downsampling, the feature maps are added to the subnetwork one by one from high resolution to low resolution, and each multiresolution feature is connected. The proposal of spectrum convolution is inspired by signal propagation. We can regard the information propagation in the convolution of spectrum diagram as the signal propagation along the nodes. Spectrum convolution uses the characteristic decomposition of Laplacian matrix of graph to realise this kind of information dissemination. Simply put, the feature decomposition of a graph can help to understand the structure of the graph and then classify the nodes of the graph. In order to solve the disadvantages caused by the imbalance of the number of samples in categories, the most commonly used solutions are as follows. (1) Repeat training for the samples that are difficult to classify or generate more head posture samples through data enhancement. (2) Expand the number of categories with fewer samples. However, both of the above will increase the extra training process and time of the model. This paper tries to alleviate the problem by improving the classification loss, which will be more convenient for model training.

## 4. Result Analysis and Discussion

In this paper, FolkDance data set and DanceDB dance video database are used to verify the dance data set. In order to see the difference and correlation between cross-entropy loss and balance loss more clearly, a set of curves of balance loss can be obtained by adjusting the nonnegative adjustment factor from 1 to 5, as shown in Figure 3.

As can be seen from Figure 3, cross-entropy loss is a special case of equilibrium loss. When the nonnegative adjustment factor is 0, the balance loss degenerates into cross-entropy loss, and the expressions of both are consistent. With the increase of nonnegative adjustment factor, the above characteristics of balance loss will become more significant. In this paper, the left-one cross-validation method is selected on the dance data set. One person's dance data set is selected as the test set, and the other three people's dance data sets are selected as the training set. The test results are shown in Figure 4.

From the data in Figure 4, it is found that as the number of people in the image increases, the time spent by this algorithm also increases gradually, but only slightly. In order to enrich the samples and improve the identification accuracy of low-resolution and blurred images by the network, two data enhancement methods are adopted for the samples used. One is to randomly flip the image left and right, which is convenient for processing and can simply get the processed body posture according to the angle of the processed body posture and is used to expand the number of samples. Another way is to blur the image locally. Considering that the actual images are often out of focus and motion blur, this paper adopts Gaussian blur and motion blur to blur the sample image locally. Comparison of F1 values of different algorithms is shown in Figure 5.

RETRACTED

After getting the binary image of the current moment of the action video, it is necessary to separate the moving region from the scene, which involves the segmentation of the moving region. In order to verify the effectiveness of this network in feature extraction of dance movements, we choose to compare it with the two methods of Inception-v3 and Fusion Inception and carry out the following ablation experiments with different feature extraction networks. Taking MSE as the evaluation index, Figure 6 shows the effectiveness test results of different networks on the test set.

The results show that the MSE of this network is obviously reduced when it is used as feature extraction network. In this paper, the network improves the accuracy of the estimation of three attitude angles. The following gives a comparison of recognition results on two data sets by extracting HOG features from the image produced by the cumulative edge feature algorithm and extracting HOG features from the original dance image.  Table 2 shows the comparison of two HOG feature recognition results on FolkDance data set.

The results in the table show that the recognition result of HOG features extracted from the accumulated edge feature images generated by the feature algorithm proposed in this paper is better than that of the traditional HOG features extracted from the original dance images.  Figure 7 shows the recognition result of the algorithm on the data set.

According to the data in Figure 7, the recognition rate of this method is the highest. A large number of experimental results in this chapter show that the algorithm proposed in this paper is 9.87% higher than *F*1 of the Incision *v*3 algorithm, and the identification accuracy is 6.51% and 10.76% higher than that of the Incision *v*3 algorithm and the traditional CNN, respectively. Through comparative experiments, it can be found that the method proposed in this paper has higher identification accuracy and faster running speed.

RETRACTED

## 5. Conclusions

The technology for estimating human posture has many applications, including dance recognition. Intelligent dance assistant training can benefit from dancers using dance recognition technology to correct poor posture. In this paper, a dance movement recognition method based on DL network is designed and proposed in accordance with the characteristics of dance movements. This paper uses Mobile Net, a thin network, as its backbone network. The two-dimensional convolution network, which can only extract spatial features, can extract and fuse time domain features by combining the time domain modelling strategy of time domain feature transfer between convolution layers and use it for dance movement recognition. This study also develops a spatiotemporal graph convolution network based on a graph transformation that can determine the relationship between any two key points of bones and improve each key point's ability to express features. The adjacency matrix can be transformed by the graph transformation module to determine the ideal graph structure. Numerous experimental findings demonstrate that the algorithm suggested in this paper is 9.87% better than *F*1 of the Incision *v*3 algorithm and that the identification accuracy is 6.51% and 10.76% better than that of the Incision *v*3 algorithm and the traditional CNN, respectively. Furthermore, the algorithm presented in this paper performs well in real time, allowing for accurate dance movement identification and correction. The work done in this paper still needs to be enhanced and deepened, though, for a number of different reasons. In the future, it will be necessary to design a more universal framework for natural human-computer interaction in the embedded mobile device environment based on the methods suggested in this paper, on the one hand, and a more lightweight and effective identification network, on the other.

## Figures and Tables

**Figure 1:** NN model.

**Figure 2:** Dance action recognition process based on DL network.

**Figure 3:** Balance loss function curves of different nonnegative adjustment factors.

**Figure 4:** Performance test results of algorithm.

**Figure 5:** Comparison of F1 values of different algorithms.

**Figure 6:** Effectiveness test results of different networks on the test set.

**Figure 7:** Recognition results of different algorithms on data sets.

**Table 1:** Basic architecture of Mobile Net network.

Input size	Module	Expansion factor	Number of channels	Layers	Step size
224^2^ × 3	conv2d 3 × 3	—	32	1	2
112^2^ × 32	Bottleneck	2	16	2	1
112^2^ × 16	Bottleneck	6	24	2	1
56^2^ × 24	Bottleneck	6	32	3	2
28^2^ × 32	Bottleneck	6	64	4	2
14^2^ × 64	Bottleneck	6	64	3	1
14^2^ × 96	Bottleneck	6	96	3	2
7^2^ × 160	Bottleneck	—	320	2	1
7^2^ × 320	conv2d 1 × 1	—	1280	1	1
7^2^ × 1280	Avgpool 7 × 7	—	—	1	—
1^2^ × 1280	conv2d 1 × 1	—	*k*	—	—

RETRACTED

**Table 2:** Comparison of different HOG feature recognition results on FolkDance data set.

Characteristic	Data set follow step double flower combination (%)	Lipian flower combination (%)	Towel flower combination (%)	Piece flower combination (%)
Traditional HOG extraction	37.98	32.14	24.13	23.41
HOG extraction in this paper	43.15	42.67	34.57	31.68
Hog extraction in literature [16]	39.17	38.87	30.75	28.81

## Data Availability

The data used to support the findings of this study are available from the corresponding author upon request.
